This article has been retracted.

# Impact of ANN in Revealing of Viral Peptides

**DOI:** 10.1155/2022/7760734

**Published:** 2022-08-08

**Authors:** M. Rajkumar, Shankar Nayak Bhukya, N. Ahalya, G. Elumalai, K. Sivanandam, Khalid M. A. Almutairi, Wadi B. Alonazi, S. R. Soma, Markos Makiso Urugo

**Affiliations:** ^1^Department of Computer Science and Engineering, Rajalakshmi Engineering College, Chennai, Tamil Nadu, India; ^2^Department of Computer Science and Engineering (Data Science), CMR Technical Campus, Hyderabad, Telangana 501401, India; ^3^Department of Biotechnology, MS Ramaiah Institute Technology, Bengaluru, Karnataka 560054, India; ^4^Department of Electronics and Communication Engineering, Panimalar Engineering College, Chennai, Tamil Nadu 600123, India; ^5^Department of Electronics and Communication Engineering, M.Kumarasamy College of Engineering, Karur, Tamil Nadu 639113, India; ^6^Department of Community Health Sciences, College of Applied Medical Sciences, King Saud University, P. O. Box: 10219, Riyadh 11433, Saudi Arabia; ^7^Health Administration Department, College of Business Administration, King Saud University, PO Box: 71115, Riyadh 11587, Saudi Arabia; ^8^Department of Biology, University of Tennessee Health Science Center, Memphis, USA; ^9^Department of Food Science and Postharvest Technology, College of Agricultural Sciences, Wachamo University, Hosaena, Ethiopia

## Abstract

All organisms contain antimicrobial peptides (AMPs), which are a critical component of the innate immune system. These chemicals have the ability to suppress the growth of a variety of fungi, bacteria, and viruses. Because AMPs interact with structural components of the microbial cell membrane and have a wide range of cellular targets, bacteria are unlikely to be able to develop resistance to them in the short term. The underlying structure of AMPs is critical in determining the selectivity with which they target their respective targets. As far as we know, peptides have not been tested in a lab to see if they can fight bacteria, fungus, and viruses in real life. In this paper, we develop an artificial neural network (ANN) using a back propagation neural network (BPNN) that enables optimal classification of tendency of a peptide sequence that involves the activities of antifungal, antibacterial, or antiviral. The BPNN is trained on the datasets collected across different repositories and then the overfitting is avoided using particle swarm optimization (PSO) algorithm. Hence, at the time of testing, the BPNN clearly finds the predicted samples belonging to the same classes and this avoids the problem of finding the false positives. The simulation is conducted to test the efficacy of the model against various metrics that includes accuracy, precision, recall, and f1-measure. The effectiveness of the BPNN-PSO model in classifying instances at a faster rate than other techniques is demonstrated by its performance. The principle is straightforward, it is not difficult to programme, it converges more quickly, and it generally offers a superior solution.

## 1. Introduction

With a collection of antimicrobial peptides (AMPs) as in Figure 1, several algorithms can predict the activity of peptide sequence using only the sequence itself. In recent years, many bioinformatics applications have demonstrated significant success when using machine learning techniques, particularly when dealing with massive volumes of biomedical information [1]. It is believed that deep learning in proteomics will become increasingly important as the big data era continues, particularly in the field of genomics. Deep neural networks with convolutional and recurrent layers are used to detect different types of peptides for HLA peptides based on the primary sequence composition of the peptides. AMPs have been the focus of multiple curated public resources, each of which provides thorough annotations based on experimental verification. This is due to the functional significance of AMPs. There are additional databases on modes of action and activities that are available to the public.

A significant number of investigations into potential cellular pathways have been made possible as a result of the discovery of AMPs [2]. An effort is being made to create computational approaches for reliably predicting AMPs in an effort to reduce the amount of time and effort required to detect AMPs experimentally [3]. As a result, AMPs computational prediction is a beneficial and supplementary method to time-consuming and labor-intensive characterisation, as it allows for the identification of possible AMP candidates that can then be tested experimentally [4–6].

Many approaches are created previously and published, and more are being developed. In terms of the approach that these tools apply, there are now two major categories of these tools [7]. Conventional machine learning-based predictors, such as the Collection of AMP, fall into the first of these two categories. They apply machine learning approaches to identify AMPs based on peptide sequence features that are determined using these tools and then identify the AMPs based on these properties [8–10].

In the field of machine learning-based predictions, the artificial neural network (ANN) is the most extensively used method, respectively [11, 12]. Deep learning-based methods are all classified as belonging to the second category. During the last few years, deep learning has become popular in bioinformatics, especially in biological sequences. For example, one-hot encoding technique is widely utilised as an input for this second class of tools. They may also combine sequence information, and they may use a neural network structure to extract features and provide classification labels, among other things. Machine learning algorithms almost never employ inputs encoded from the original sequences as inputs to their computations.

Machine learning can uncover the knowledge of sequences by comparing known sequences of AMP to unknown AMP sequences in a database. Machine learning can be used to investigate the physicochemical mechanisms of membrane permeability since it is capable of measuring the key properties of peptides that allow them to penetrate membrane barriers [13, 14].

When it comes to learning methods that do not require direct instruction, unsupervised approaches are quickly gaining ground in the growing amount of research on the subject. The majority of the approaches described in this research are based on supervised learning on well-tested AMP datasets. The number of annotated AMPs continues to grow, which has resulted in the development of novel computations. Furthermore, these methods involve feature estimation and selection algorithms in addition to the more traditional machine learning-based methodologies. There is an urgent need for new and improved ways to address the problem of high false-positive rates, which plague the bulk of current treatments and which must be addressed immediately.

An artificial neural network approach that permits optimal categorisation of a peptide sequence potential to have antifungal, antibacterial, or antiviral activity has been developed in this research, which makes use of a back propagation neural network (BPNN). A strategy known as particle swarm optimization (PSO) prevents overfitting by training the BPNN.

## 2. Literature Survey

Because of the large number of AMP sequences and structures available, as well as the time and resources required to develop, manufacture, and test potential AMP candidates, it is not possible to screen the whole peptide sequence space experimentally. It can be time-consuming and expensive to calculate and measure molecular activity. Therefore, QSAR models aim to harness physical and chemical properties to predict biological activity. A peptide sequence, on the other hand, can be used to compute many of its physical and chemical properties [15, 16] without requiring significant computational resources.

A wide variety of statistical learning methods have been employed in the construction of QSAR models for the purpose of computational amplifier design. For the first time, AMP classification tools based on QSAR were developed by [17] in their research of the C and N-terminal residues. They [18] trained an ANN using the antibacterial efficacies and tested against various bacteria resistant.

With the help of HMMs, [19] found a hitherto undiscovered AMP in the bovine genome and proved that the bovine genome did not contain -defensins, which were previously thought to be present. In 2009, this group utilised a similar strategy to uncover 18 synthetic AMP sequences with high antibacterial action against multidrug-resistant bacteria [15], which was published in Nature Chemical Biology. In another study [20], AMPs were classified with 75–90% accuracy using an eight-descriptor support vector machine trained to categorise AMPs while taking novel factors such as peptide aggregation into account.

A two-level classifier developed by [21] was used to first categorise peptide sequences and classify into groups based on their structural characteristics. They [22] used graph theory that included many bioactivity markers, in order to recommend new candidates for clinical trials in 2015.

They [23] used unsupervised–supervised two-step models for the first time to categorise AMPs, which was a first in the field. They applied nonlinear dimensionality reduction to the training data by employing self-organising maps, and the resulting data was then put into a supervised neural network model for classification. According to the findings of these investigations, a diverse range of methodologies and approaches have been successfully employed in the classification and construction of AMPs.

## 3. Proposed Method

A back propagation neural network (BPNN) is used in this paper to construct an artificial neural network framework that helps optimal categorisation of a peptide sequence's potential to have antifungal, antibacterial, or antiviral activity. The core of the neural network training process is called back propagation. The process of fine-tuning the weights of a neural net depending on the error rate achieved in the previous epoch is referred to as the practice of back propagation of errors. The entirety of the AVP model that was proposed includes multiple stages, including preprocessing, feature extraction, BPNN-PSO Classification, and finally the prediction, which is revealed in the AVP concept aspect that is displayed in Figure 2.

### 3.1. Feature Extraction

Peptide sequences must first be transformed into numeric feature vectors before they can be used as input for a machine learning classifier. It makes use of iFeature, a tool that can calculate and analyse a large number of features, develop ML models, and classification issues involving protein sequence, DNA, and RNA. iFeature is a powerful tool that can calculate and analyse a large number of features, develop machine learning models, and evaluate their performance.

In order to limit the number of features to 100, the feature selection methods available in iFeature use information gain. Following the construction of these predictions, the BPNN was used to compare their performance to that of the other forecasts. A 5-fold cross-validation approach was used to evaluate all of the models in this study.

### 3.2. Classification

Training the BPNN, which is a feed-forward network with multiple layers, is accomplished by the use of an error-back propagation method. BPNN is capable of performing a large number of input-output mappings without having to know the actual mathematical equations underlying them. After the network parameters have been adjusted for all inputs, gradient descent allows the network to continue to adjust them during the error propagation process.

A BPNN is comprised of multiple levels of the network. However, a three-layer BPNN is typically deemed sufficient for approximating the mapping relationships between inputs and outcomes in mathematical equation models, as shown in the following example. Accordingly, the usual BPNN structure is composed of three layers: the input layer, one hidden layer, and the output layer. Let **s** represent a single input instance and **n** represent the number of inputs in the input layer.

(1) $$\begin{array}{c} s=\left\{a_{1},a_{2},a_{3},\cdots ,a_{n}\right\}, \end{array}$$

*w*_*ij*_ - weight assigned to each input to a neuron,

**j** - input (source and destination nodes).

The **j**^th^ neuron in a layer has an optional parameter *θ*_*j*_, which is a bias that can be used to change the activity of the neuron. The default value for this parameter is 1.

The output of the preceding neuron is denoted by *o*_*j*_, and the input *I*_*j*_ of the following neuron can be calculated using Eq (2).

(2) $$\begin{array}{c} I_{j}=\underset{i}{\sum }w_{ij}o_{j}+\theta_{j}. \end{array}$$

Sigmoid functions are widely employed to determine the output of neurons *o*_*j*_; consequently, Eq. (3) can be used to obtain the neuron output from the sigmoid function.

(3) $$\begin{array}{c} o_{j}=\frac{1}{1+e^{-I_{j}}}. \end{array}$$

As soon as the feed-forward procedure is completed, the reverse propagation process begins.

Let *Err*_*j*_ be the error sensitivity of a neuron **j** in the output layer, and let *t*_*j*_ denote the desired output of a neuron **j** in the output layer, as follows (4):

(4) $$\begin{array}{c} {Err}_{j}=o_{j}\left(1-o_{j}\right)\left(t_{j}-o_{j}\right). \end{array}$$

With *Err*_*k*_ representing a neuron error sensitivity and *w*_*kj*_ representing its weight, Eq. (5) may be used to compute *Err*_*j*_ for the neuron in the following layer by utilising *Err*_*k*_ and *w*_*kj*_, respectively (5).

(5) $$\begin{array}{c} {Err}_{j}=o_{j}\left(1-o_{j}\right)\underset{k}{\sum }{Err}_{k}w_{kj}. \end{array}$$

As a result, by modifying the weights and biases of each neuron during the back propagation process, Eqs. (6)–(9) can be used to alter the learning rate **η** of the network.

(6) $$\begin{array}{c} ∆w_{ij}={Err}_{j}o_{j}, \end{array}$$

(7) $$\begin{array}{c} w_{ij}=w_{ij}+\eta ∆w_{ij}, \end{array}$$

(8) $$\begin{array}{c} ∆\theta_{j}={Err}_{j}, \end{array}$$

(9) $$\begin{array}{c} \theta_{j}=\theta_{j}+\eta ∆\theta_{j}, \end{array}$$

Following the tuning of the network parameters by one input instance, BPNN begins to input the next instance into the network. BPNN does not complete its training phase until either Eq. (10) or Eq. (11) for a single output or multiple outputs are met.

(10) $$\begin{array}{c} \min\left(E\left[e^{2}\right]\right)=\min\left(E\left[{\left(t-o\right)}^{2}\right]\right), \end{array}$$

(11) $$\begin{array}{c} \min\left(E\left[e^{T}e\right]\right)=\min\left(E\left[{\left(t-o\right)}^{T}\left(t-o\right)\right]\right). \end{array}$$

In order to classify data, only the feed forward is required. The results of the classification are displayed in the output layer.

### 3.3. Overfitting

A wide range of applications have been improved as a result of the use of PSO algorithms. PSO works by placing all individuals and particles in the search space at random, which is how it operates. The particles then move in a random direction inside the search space, with each particle moving in a different direction every time. Next, it is necessary to recalculate each particle route, taking into account its previous movements and the most advantageous locations it has already visited. This process is repeated for each new particle (i.e., fitness). Particle speed and position are picked at random, and the results are used to generate updates to the velocity formula, which is illustrated below:

(12) $$\begin{array}{c} {Vc}_{i+1}=wV_{i}+C1R1\times \left({Pb}_{i}-x_{i}\right)+C2R2\times \left(Gb-x_{i}\right). \end{array}$$

In contrast, the velocity of the new particle is added to the velocity of the preceding particle to provide the following result:

(13) $$\begin{array}{c} x_{i+1}=x_{i}+{Vc}_{i+1}, \end{array}$$

where

*Vc* - particle velocity

**x** - particle position

*R*_1_ and *R*_2_ - random variables distributed as [0, 1]

*C*_1_ and *C*_2_ - acceleration coefficients and

**w** - inertia weight

Obtaining the particle new velocity requires knowledge of the particle previous velocity, its current position relative to its ideal position (Pb), and the best position available everywhere on the globe (GB). Each particle is assigned a new location in the search space in accordance with the results of Eq. (3), which is based on the performance index. This means that each particle is evaluated in relation to an objective function that has been established. The proposed methodology adjusts the architecture, synaptic weights, and type of transfer functions of BPNNs at the same time in order to produce BPNNs that are the most accurate for a certain task.

While developing and optimising the accuracy of a BPNN, the set of transfer functions (TF), the set of synaptic weights, and biases (and their combinations) are the most important aspects to consider while developing and optimising the accuracy of a BPNN. Each of these elements should be included in the person who represents the answer to our problem. The fitness function will be used to evaluate the output of the bioinspired algorithms in order to determine the best candidate to represent the best BPNN in the final analysis. The proposed method will only be used to solve pattern categorisation problems and nothing else.

To put the technique through its paces, three particle swarm algorithms and eight fitness functions are used. A detailed behavioral examination of each algorithm must be performed as a result of this. Aside from that, the maximum number of neurons that can be generated by the technology used to construct the BPNN should be considered because it has a direct impact on the size and shape of the individual. The fact that supervised learning requires just input and output patterns to determine the size of an individual for a certain job necessitated the development of an equation that would allow us to construct the BPNN.

As illustrated in Figure 3, the recommended technique is depicted as a flowchart. In order to evaluate each individual during the training phase, it is necessary to establish the individuals and their fitness duties early on. The size of an individual psyche is influenced by the size of their input patterns as well as the size of their desire patterns. For an extended period of time, the individual will be transformed in order to come up with the best possible solution to the problem (with a minimum error). At the conclusion of the process, it is anticipated that the ANN will be able to perform admirably throughout training and testing.

## 4. Results and Discussions

The result was accomplished using a laptop equipped with an i5 processor, 8 gigabytes of random access memory (RAM), and a processing speed of 2.8 gigahertz, which was run on a computer system. We were able to conduct data analysis by using a Python notebook on which all of the relevant libraries had been pre-installed. This allowed us to perform tasks such as model development and correlation analysis. In this part of the study, the DRAMP 2.0 datasets are utilised so that the effectiveness of our ANN-PSO approach may be evaluated. For starters, we will evaluate the performance of numerous modules in order to determine how trustworthy our strategy is. The study puts ANN approach to the test against the approaches of using a well-researched dataset, and the results were overwhelmingly positive. Because some of the training datasets for the tools we examined are no longer available, and because the training datasets for several other tools have been increased, however, there exists an overlap between the used datasets for the generation of tools to generate the independent dataset.  Table 1 shows accuracy of various models along with the proposed approach.

A role for the training set may be seen in the gap between the predictions made by the different methodologies (Figures 4–7). First, cross-validation was used to compare the performance of the classic machine learning algorithms against one another. CD-HIT was utilised to identify and remove redundant information from the positive samples from AMP datasets, which was then analysed further.

## 5. Discussion

AMPs with specific functional effects are well-known, and this has sparked the interest of biologists who are interested in learning more about them. AMPs having a wide range of functionalities are overrepresented, resulting in an uneven distribution of computational workload. Because of this, it is extremely difficult to predict the exact roles of AMPs in advance. The majority of computer techniques are now centered on AMP prediction. As a result of the distinct sequences and secondary structures of AMPs, as well as their physical and chemical properties, there will be a wide range of predictability issues depending on their function. Because of this, we evaluated the predictive capacities of several approaches and compared the variance in prediction accuracy among them.

Initially, the study identifies the total AMPs found in the sample that were used for a variety of functions. The BPNN-PSO method was proven to be the most accurate method for determining if AMPs possessing anticancer, antibacterial, antitumor, antifungal, or antiviral properties are in fact AMPs. In terms of prediction performance, SVM outperformed the competition for AMPs with antibiofilm action.

When it came to discovering antifungal, antibacterial, and antiviral AMPs, the PSO-BPNN technique performed admirably. Among the other methods tested, BPNN-PSO and SVM proved to be the most accurate in predicting AMPs with insecticidal capabilities, as did other approaches.

The highest accuracy of BPNN was achieved through the selection of features based on mutual information. The use of feature selection allowed for the highest accuracy score to be reached. When the information gain is used, the BPNN-PSO model proved to be the most accurate. It makes little difference which feature selection technique is employed as long as the AMP prediction results are competitive, if not the best, in the industry.

## 6. Conclusions

By analysing its biochemical properties, the BPNN artificial neural network approach, which we offer in this research, can be used to detect the antifungal, antibacterial, and antiviral effects of aAMP. The BPNN is trained using data from many repositories, and it is then safeguarded from overfitting using the PSO approach, which is based on the principle of least squares. Because the BPNN locates predicted samples that belong to the same class at the time of testing, the problem of false positives is eliminated. As part of the simulation, the model is assessed against a variety of metrics, including accuracy, precision, recall, and f1-measurement, among others. The performance of the BPNN-PSO model demonstrates that it is more effective than other methods at classifying instances at a faster rate than other methods. On the basis of certain common features extracted from sequences in this investigation, preliminary comparisons of prediction outcomes from numerous classic ML models, as well as a preliminary assessment of the significance of certain aspects, were made in this work.

ML-based techniques can benefit from a variety of different strategies that can assist them in becoming more accurate forecasters of the future. The technique has recently acquired popularity as a ML model, and it has also garnered traction in related fields such as bioinformatics and computational biology. Despite the fact that deep learning frameworks are utilised in a variety of methods to detect AMPs, the deep learning structures of these frameworks are easy. In the future, the improvement can be achieved more effectively than with other methods already in use by using a number of other deep learning algorithms.

## Figures and Tables

**Figure 1:** AMP classes.

**Figure 2:** Proposed AVP model.

**Figure 3:** Proposed training and testing model.

**Figure 4:** Accuracy.

**Figure 5:** Precision.

**Figure 6:** Recall.

**Figure 7:** F-measure.

**Table 1:** Accuracy of various models along with proposed approach.

Model	Accuracy (%)
KNN	79
K means	87
SVM	90
BPNN	93
BPNN-PSO	98

## Data Availability

The data used to support the findings of this study are included within the article. Further data or information is available from the corresponding author upon request.
